This article has been retracted.

# MicroRNA-300 inhibited glioblastoma progression through ROCK1

**DOI:** 10.18632/oncotarget.9068

**Published:** 2016-04-28

**Authors:** Fucheng Zhou, Yang Li, Zhen Hao, Xuanxi Liu, Liang Chen, Yu Cao, Zuobin Liang, Fei Yuan, Jie Liu, Jianjiao Wang, Yongri Zheng, Deli Dong, Shan Bian, Baofeng Yang, Chuanlu Jiang, Qingsong Li

**Affiliations:** ^1^ Department of Neurosurgery, The 2nd Affiliated Hospital, Harbin Medical University, Harbin 150086, China; ^2^ Harbin Medical University, Harbin 150086, China; ^3^ Institute of Molecular Biology, Austrian Academy of Sciences, Vienna, Austria

**Keywords:** glioblastoma, microRNAs, miR-300, ROCK1

## Abstract

Glioblastoma is a common type of brain aggressive tumors and has a poor prognosis. MicroRNAs (miRNAs) are a class of small, endogenous and non-coding RNAs that play crucial roles in cell proliferation, survival and invasion. Deregulated expression of miR-300 has been studied in a lot of cancers. However, the role of miR-300 in glioblastoma is still unknown. In this study, we demonstrated that miR-300 expression was downregulated in glioblastoma tissues compared with the normal tissues. Lower expression level of miR-300 was observed in thirty cases (75 %, 30/40) of glioblastoma samples compared with the normal samples. Moreover, the overall survival of glioblastoma patients with lower miR-300 expression level was shorter than those with higher miR-300 expression level. In addition, miR-300 expression was also downregulated in glioblastoma cell lines. Overexpression of miR-300 inhibited cell proliferation, cell cycle and invasion in glioblastoma cell line U87 and U251. Moreover, we identified ROCK1 as a direct target of miR-300 in U87 and U251 cells. Overexpression of ROCK1 partially rescued the miR-300-mediated cell growth. ROCK1 expression levels in glioblastoma tissues were higher than that in normal tissues. ROCK1 expression levels were higher in thirty-one cases of glioblastoma samples than their normal samples. Furthermore, the expression level ROCK1 was inversely correlated with the expression level of miR-300. Importantly, overexpression of miR-300 suppressed glioblastoma progression in an established xenograft model. In conclusion, we revealed that miR-300 might act as a tumor suppressor gene through inhibiting ROCK1 in glioblastoma.

## INTRODUCTION

Glioblastoma is a common form of primary malignant brain tumors and the 5-year survival rate is less than 3% [1–3]. Glioblastoma is characterized by high infiltrative invasion and proliferation [4–8]. Despite the combined treatment with chemotherapy, radiotherapy and surgery, the overall survival of glioblastoma patients is just about 1 to 2 years [9–12]. Therefore, it is crucial to identify novel effective therapeutic targets to reduce glioblastoma mortality.

MicroRNAs (miRNAs) are a class of small (approximately 22 bases), single-stranded and non-coding RNAs that bind to the complementary sites in 3′untranslated regions (3′-UTR) of target genes to induce translational repression or degradation [13–17]. Increasing studies have showed that miRNAs play pivotal roles in cell proliferation, metabolism, differentiation, invasion and migration [18–24]. More importantly, miRNAs play important roles in cancer progression and initiation and function as tumor suppressors or oncogenes [25–27]. Abnormal expressions of miRNAs are associated with various cancers such as gastric cancer, renal cell carcinoma, breast cancer, ovarian carcinoma and osteosarcoma [28–32].

In the present study, we showed that miR-300 expression was downregulated in glioblastoma tissues and cell lines. Moreover, lower expression of miR-300 was correlated with shorter survival in glioblastoma. Furthermore, miR-300 suppressed cell proliferation and invasion by inhibiting ROCK1 in glioblastoma cells.

## RESULTS

### MiR-300 expression was downregulated in glioblastoma cell lines and tissues

MiR-300 expression was downregulated in glioblastoma tissues compared with their normal tissues (Figure 1A and 1B). In general, the expression of miR-300 in glioblastoma tissues was lower than in normal tissues (Figure 1C). Among 40 cases, thirty cases (75 %, 30/40) showed lower level of miR-300 in glioblastoma samples compared with their normal samples (Figure 1D). The overall survival of glioblastoma patients with low miR-300 expression was lower than those with high expression (Figure 2A). In addition, miR-300 expression was downregulated in glioblastoma cell lines (U87, U373, U251 and A172) than in NHAs (Figure 2B).

**Figure 1:** The expression of miR-300 was down-regulated in glioblastoma tissues **A, B.** The expression of miR-300 in glioblastoma tissues was measured by using qRT-PCR. **C.** The expression of miR-300 in glioblastoma tissues was significant lower than in normal tissues. **D.** Thirty cases (75 %, 30/40) showed lower level of miR-300 in glioblastoma samples compared with their normal samples.

**Figure 2:** The expression of miR-300 was down-regulated in glioblastoma cell lines **A.** The overall survival of glioblastoma patients with low miR-300 expression was lower than that of patients with high expression. **B.** The expression of miR-300 in glioblastoma cell lines and NHAs was measured by using qRT-PCR.

### MiR-300 inhibited glioblastoma cell proliferation, cell cycle and invasion

MiR-300 mimic was transfected into U87 and U251 cells and the efficiency of miR-300 was confirmed by qRT-PCR analysis (Figures 3A and 3B). Overexpression of miR-300 inhibited the cell proliferation in U87 and U251 cells (Figures 3C and 3D). Furthermore, ectopic expression of miR-300 repressed cell cycle in U87 and U251 cells (Figures 3E and 3F). In addition, ectopic expression of miR-300 inhibited cell invasion in U87 and U251 cells (Figures 3G and 3H).

**Figure 3:** miR-300 inhibited glioblastoma cell proliferation, cell cycle and invasion **A, B.** The expression of miR-300 in U87 and U251 cells was detected by using qRT-PCR. **C, D.** The cell proliferation was measured by using CCK-8 assay in U87 and U251 cells. **E, F.** ectopic expression of miR-300 repressed the U87 and U251 cells cycle. **G, H.** ectopic expression of miR-300 repressed the U87 and U251 cells invasion. *p<0.05, and **p<0.01, *** p<0.001.

### ROCK1 was the direct target of miR-300

Bioinformatic analysis showed that the 3′UTRs of ROCK1 had at least 7 nucleotides that were complementary to the miR-300 seed region (Figure 4A). We integrated a fragment of the ROCK1 3′UTR containing a fragment whose target site was mutated, into a luciferase reporter vector (Figure 4B). Overexpression of miR-300 inhibited the luciferase activity of Wt-3′UTR of ROCK1 by about 60% compared with the mutated miR-300 binding site (Figures 4C and 4D). Ectopic expression of ROCK1 suppressed ROCK1 expression in U87 and U251 cells (Figures 4E and 4F).

**Figure 4:** ROCK1 is the direct target of miR-300 **A, B.** The WT and Mut of 3′UTR of ROCK1 mRNA contains the binding sequences of miR-300. **C, D.** Relative luciferase activity of the indicated PDK1 reporter construct in U87 and U251 cells is shown. Firefly luciferase values were normalized to Renilla luciferase activity and plotted as relative luciferase activity. **E, F.** The protein expression of ROCK1 in U87 and U251 cells was measured by western blot. *** p<0.001.

### Overexpression of ROCK1 partially rescued the miR-300-mediated cell growth

The efficiency of ROCK1 vector was confirmed by western blot and qRT-PCR analysis (Figures 5A and 5B). CCK8 analysis demonstrated that ectopic expression of ROCK1 partially rescued the miR-300-mediated cell growth in U87 and U251 cells (Figures 5C and 5D). Furthermore, the cell cycle arrest overexpressing miR-300 was partially increased after transfection of ROCK1 vector (Figures 5E and 5F).

**Figure 5:** Overexpression of ROCK1 partially rescued the miR-300-mediated cell growth **A.** The protein expression of ROCK1 in U87 cells was measured by western blot. **B.** The mRNA expression of ROCK1 in U87 cells was measured by qRT-PCR. **C, D.** The cell proliferation was measured by using CCK-8 assay in U87 and U251 cells. **E, F.** The cell cycle was detected by using flow cytometry. *p<0.05, and **p<0.01, *** p<0.001.

### The expression level of ROCK1 was inversely correlated with the expression level of miR-300

The expression of ROCK1 in glioblastoma tissues was higher than in normal tissues (Figure 6A). Thirty-one cases (78 %, 31/40) showed higher level of ROCK1 in glioblastoma samples compared with their normal samples (Figure 6B). Furthermore, ROCK1 expression level was inversely correlated with the expression level of miR-300 (r2=−0.279; p<0.001) (Figure 6C).

**Figure 6:** The expression of ROCK1 was inversely with the expression of miR-300 **A.** The expression of miR-300 in glioblastoma tissues was significant lower than in normal tissues. **B.** Thirty-one cases (78 %, 31/40) showed higher level of ROCK1 in glioblastoma samples compared with their normal samples. **C.** The ROCK1 expression was inverse correlated with the expression of miR-300 (r=−0.528; p<0.001).

### MiR-300 inhibited the growth of U87-engrafted tumors

We confirmed that miR-300 mimics enhanced the expression of miR-300 in the U87-engrafted tumors (Figure 7A). MiR-300 mimics suppressed the growth of U87-engrafted tumors compared with scrambled oligonucleotides-treated tumors (Figure 7B). Moreover, the weights of tumors treated by miR-300 were lower than the scrambled-injected tumors (Figure 7C). Injection of miR-300 mimic inhibited the growth of U87-engrafted tumors compared with the scrambled oligonucleotides-treated tumors (Figure 7D). ROCK1 expression was lower in miR-300-treated tumors compared with the scramble-treated tumors (Figures 7E and 7F).

**Figure 7:** miR-300 inhibited the growth of U87-engrafted tumors **A.** The expression of miR-300 was measured by qRT-PCR. **B.** We demonstrated that miR-300 mimic suppressed the growth of U87-engrafted tumors compared to scrambled oligonucleotides-treated tumors. **C.** The weights of tumors treated by miR-300 were lower than scrambled-injected tumors. **D.** Representative tumors were photographed treatment with miR-300 mimic or scramble. **E.** The mRNA expression of ROCK1 was measured by qRT-PCR. **F.** The protein expression of ROCK1 was measured by western blot. *p<0.05, and **p<0.01, *** p<0.001.

## DISCUSSION

In this study, we demonstrated that miR-300 expression was downregulated in glioblastoma tissues compared with their normal tissues. Thirty cases (75 %, 30/40) of total patients showed lower level of miR-300 in glioblastoma samples compared with their normal samples. The overall survival of glioblastoma patients with low miR-300 expression was lower than those with high expression. In addition, miR-300 expression was downregulated in glioblastoma cell lines. Overexpression of miR-300 inhibited cell proliferation, cell cycle and invasion in U87 and U251. We identified ROCK1 as a direct target of miR-300 in U87 and U251 cells. Overexpression of ROCK1 partially rescued the miR-300-mediated cell growth. Moreover, the expression level of ROCK1 in glioblastoma tissues was higher than in normal tissues. Thirty-one cases of total patients showed increased level of ROCK1 in glioblastoma samples compared with their normal samples. Furthermore, ROCK1 expression level was inversely correlated with the expression level of miR-300. Importantly, overexpression of miR-300 suppressed progression of glioblastoma in an established xenograft model. These data suggested that miR-300 played an important role in inhibiting the progression and development of glioblastoma.

Recent studies have demonstrated that miR-300 plays important roles in tumor development [33–35]. For example, Zhang et al. showed that miR-300 was commonly upregulated in glioma tissues, and the expression of miR-300 was higher in glioma stem-like cells (GSLCs) [36]. Moreover, miR-300 enhanced the GSLCs self-renewal and reduced differentiation by inhibiting LZTS2 expression. Xue et al. found that miR-300 expression was increased in osteosarcoma cell lines and tissues [37]. Overexpression of miR-300 increased osteosarcoma cell invasion, proliferation and EMT by inhibiting bromodomain-containing protein 7 (BRD7) expression. In this study, we found that miR-300 expression was downregulated in glioblastoma tissues compared with their normal tissues. The overall survival of glioblastoma patients with low miR-300 expression was lower than that of patients with high expression. In addition, miR-300 was downregulated in glioblastoma cell lines. Overexpression of miR-300 inhibited cell proliferation, cells cycle and invasion in U87 and U251 cells. We also found that overexpression of miR-300 suppressed progression of glioblastoma in an established xenograft model. The contrasting data may be due to the indistinctive change and the different quantity of clinical samples.

MiRNAs play their roles through binding to their target mRNAs and inhibiting their protein expressions [38–40]. In our study, we identified ROCK1 as a direct target of miR-300 in glioblastoma. TargetScan and dual luciferase activity assay showed that there was a putative-binding site on the 3′UTR of ROCK1 mRNA with miR-300. Overexpression of miR-300 suppressed the luciferase activity of reporter vector with miR-300 response elements. Ectopic expression of miR-300 inhibited the expression of ROCK1 in both U87 and U251 cells. More importantly, we found that overexpression of ROCK1 partially rescued the miR-300-mediated cell growth. We also demonstrated that the expression level of ROCK1 in glioblastoma tissues was higher than in normal tissues. In addition, the ROCK1 expression level was inversely correlated with the expression level of miR-300 in glioblastoma tissues. These data suggested that miR-300 inhibited glioblastoma cell proliferation, cell cycle and cell invasion through suppressing ROCK1.

In summary, we showed that miR-300 was downregulated in glioblastoma tissues and cell lines. Moreover, low expression of miR-300 was correlated with short survival in glioblastoma patients. We demonstrated that miR-300 suppressed cell proliferation and invasion by suppressing ROCK1 in glioblastoma cells. In conclusion, we revealed that miR-300 might act as a tumor suppressor gene through inhibiting ROCK1 in glioblastoma.

## MATERIALS AND METHODS

### Patient samples and cell lines

Human glioblastoma samples and non-neoplastic samples (located >3 cm from the tumors) were taken from our hospital. These patients had not received radiotherapy or chemotherapy before surgery. These samples were stored in liquid nitrogen until used. Human glioblastoma cell lines (U87, U373, U251 and A172) and normal human astrocytes (NHAs) were from the ATCC and cultured in DMEM/F-12 supplemented with FBS (fetal bovine serum). All Patients were given informed consent and our study was approved by the ethical board of the institute of The 2nd Affiliated Hospital of Harbin Medical University and complied with Declaration of Helsinki.

### Cell transfection

MiR-300 mimics and scramble oligonucleotides (10nmol/l), ROCK1 vector and control vector were obtained from Ambion (Ambion, USA). Cell transfection was performed using Lipofectamine 2000 (Life Technologies, USA) according to manufacturer's information.

### QRT-PCR

Total RNA extraction was performed used Trizol (Invitrogen). The relative expression of ROCK1 and miR-300 were detected using Quantitative RT-PCR (qRT-PCR) on IQ5 Real-Time PCR system and snRNA U6 or GAPDH was used as control. Primers used for miR-XX and are as follows: ROCK1, 5′-AGGA AGGCGGACATATTAGTCCCT-3′ (forward), 5′-AGAC GATAGTTGGGTCCCGGC-3′ (reverse); GAPDH, 5′-AT GTCGTGGAGTCTACTGGC-3′ (forward), 5′-TGACCTT GCCCACAGCCTTG-3′ (reverse).

### Dual luciferase activity assay

The 3′UTR target site was generated by PCR and the luciferase reporter constructs with the ROCK1 3′UTR carrying a putative miR-300-binding site into pMiR-report vector were amplified by PCR. Cells were co-transfected with the reporter construct, control vector and miR-300 or scramble using Lipofectamine 2000 (Life Technologies, USA). Reporter assays were done using the dual-luciferase assay system (Promega) following to the manufacturer's information.

### Western blot analysis

Protein from cells or tissues was extracted using BCA kit. Protein was separated by 10% SDS–PAGE and then transferred onto PVDF membranes (Millipore Corporation, USA). The membrane was blocked with 5% milk and then incubated with primary antibodies (ROCK1, GAPDH, Cell Signaling Technology, USA). The membranes were incubated with the second antibodies and then measured using the ECL detecting system (Thermo Scientific, USA). GPADH was used as loading control.

### Cell proliferation and invasion assays

Cell growth was measured by using CCK-8 assay (Dojindo, Kumamoto, Japan) according to manufacturer's information. Proliferation rate was measured at 0 hour, 24 hour, 48 hour and 72 hour after treatment. For cell invasion assay, cell was determined using Matrigel Invasion Chambers (BD Biosciences). Cells were cultured in Matrigel-coated transwell chambers and medium containing 5% FBS in the lower chamber as the chemoattractant. Invasive cells located on the lower surface of the chamber were stained with crystal violet and counted.

### In vivo tumorigenesis assay

U87 cells (5×106 cells per mouse) were inoculated subcutaneously into the dorsal flanks of 6-week-old female nude mice. On the day 10, when tumors reached about 50 mm^3^, miR-300 mimics or the scrambled (100 nmol per mouse in 100 μl total volume containing 10 μl Lipofectamine 2000and 90 μl phosphate-buffered saline) were injected into the tumors with 26-gauge needles every three days. The tumor length, width and weight were detected every 3 days. Mice were euthanized using cervical dislocation on the 25th days after cancer cell inoculation.

### Statistical analysis

Data are showed as the mean ± SD (standard deviation). The differences between groups were measured using Student t test or one-way ANOVA. Survival rate was estimated with the use of the Kaplan-Meier method. Spearman's coefficient of correlation was performed to detect the correlation. p<0.05 was considered as statistically significant.
